# LncXIST Facilitates Iron Overload and Iron Overload-Induced Islet Beta Cell Injury in Type 2 Diabetes through miR-130a-3p/ALK2 Axis

**DOI:** 10.1155/2022/6390812

**Published:** 2022-06-09

**Authors:** Weiyuan Li, Qiu Feng, Chenrong Wang, Zhao Yin, Xiaolu Li, Lei Li

**Affiliations:** ^1^Department of Geriatrics, The First People's Hospital of Yunnan Province, The Affiliated Hospital of Kunming University of Science and Technology, Kunming, Yunnan, China; ^2^Medical Laboratory, The First People's Hospital of Yunnan Province, The Affiliated Hospital of Kunming University of Science and Technology, Kunming, Yunnan, China; ^3^Department of Endocrine, The First People's Hospital of Yunnan Province, The Affiliated Hospital of Kunming University of Science and Technology, Kunming, Yunnan, China

## Abstract

Iron overload is directly associated with diabetes mellitus, loss of islet beta cell, and insulin resistance. Likewise, long noncoding RNA (lncRNA) is associated with type 2 diabetes (T2D). Moreover, lncRNAs could be induced by iron overload. Therefore, we are going to explore the molecular mechanism of lncRNA XIST in iron overload-related T2D. Real-time quantitative PCR and Western blot were used to detect gene and protein levels, respectively. TUNEL and MTT assay were performed to examine cell survival. The glucose test strip, colorimetric analysis kit, ferritin ELISA kit, and insulin ELISA kit were performed to examine the levels of glycolic, iron, and total iron-binding capacity, ferritin, and insulin in serum. Fluorospectrophotometry assay was used to examine labile iron pool level. XIST was higher expressed in T2D and iron overload-related T2D rat tissues and cells, and iron overload-induced promoted XIST expression in T2D. Higher XIST expression was associated with iron overload in patients with T2D. Knockdown of XIST alleviated iron overload and iron overload-induced INS-1 cells injury. Further, we found that XIST can sponge miR-130a-3p to trigger receptor-like kinase 2 (ALK2) expression. Moreover, knockdown of ALK2 alleviated iron overload and iron overload-induced INS-1 cells injury by inhibiting bone morphogenetic protein 6 (BMP6)/ALK2/SMAD1/5/8 axis but reversed with XIST upregulation, which was terminally boosted by overexpression of miR-130a-3p. XIST has the capacity to promote iron overload and iron overload-related T2D initiation and development through inhibition of ALK2 expression by sponging miR-130a-3p, and that targeting this axis may be an effective strategy for treating patients with T2D.

## 1. Introduction

Type 2 diabetes (T2D) is a metabolic disease mediated by environmental and genetic factors, accounting for more than 90% of the total prevalence of diabetes, and is associated with increased risk of colon, uterine, liver, pancreatic, breast (in postmenopausal women), and prostate cancers amongst others [1]. At present, it is generally believed that dysfunction and insulin resistance (IR) of *β*-cell of the pancreatic islet are two important factors in the pathogenesis of T2D pathophysiology [2]. Since 1865, it was found that the risk of T2D increases in patients with hemochromatosis [3]. The association between iron overload and T2D has been paid more attention. Histopathological and clinical findings in earlier research provide evidence that iron overload impacts the pancreatic *β*-cell and affects insulin secretion, finally leading to diabetes [4]. Subsequently, a considerable number of studies have found that the majority of patients with T2D or T1D or gestational diabetes mellitus have dysmetabolic iron [5, 6]. Hepcidin, a 25-amino acid peptide produced by the hepatocytes, is a key regulator of iron metabolism and responsible for iron deposition [7], which is dysregulated in diabetic patients. Iron overload exhibits loss of *β*-cell mass and increases hepatic glucose production and metabolic inflexibility [8, 9]. The subsequent loss of islet *β*-cell can then lead to a gradual loss of functional capacity and decreased insulin sensitivity [10, 11]. Recently, research demonstrated the association of iron homeostasis with IR in high-fat feeding mice [12]. However, the mechanism underlying the facilitation of iron on the development of T2D is still unknown.

Long noncoding RNA (lncRNA) is longer than 200 nucleotides, lacking defined protein coding potential. LncRNAs have emerged as key components of regulatory genome organization and gene expression. It is increasingly recognized that lncRNAs play an important function in the epigenetic processes in both health and disease [13, 14]. In recent years, lncRNAs are considered to be regulatory molecules in islet function and the etiology of diabetes, such as lncHI-LNC25 [15], lncH19 [16], and lncMALAT1 [17]. Moreover, altered lncRNAs signatures are found in T2D patients, including increasing expression levels of XIST [18] in PBMCs from T2D patients compared to control subjects. Besides, XIST is linked with IR and inflammation in T2D [18], also participating in diabetic cardiomyopathy [19] and diabetic nephropathy [20]. In addition, lncRNAs also mediate intracellular iron metabolism. PVT1 influenced the uptake level of cellular iron in hepatocellular carcinoma, and its upregulation induced an iron metabolism disorder and promoted tumorigenesis [21]. The relationship between XIST and iron overload in T2D is not well known.

In this paper, we have proposed a novel approach and verified its applicability through various experiments. The results showed that XIST overexpression in iron overload rats was associated with a coincident alteration in iron-related parameters. *In vitro*, increasing XIST level in response to iron-induced was associated with iron metabolism, proliferation inhibition, apoptosis, and reduction of insulin secretion. In contrast, XIST knockdown alleviated above islet *β*-cell damage induced by iron overload.

The remaining paper is organized as follows.

In the subsequent section, various groups of animals, which are formed to verify the operational superiority of the proposed scheme, are described along with various metrics. Moreover, treatment methods were described along with feasible duration. In Section 3, performance evaluation of the proposed scheme in terms of various metrics has been presented. Finally, summary of the proposed approach is presented in the conclusion section.

## 2. Materials and Methods

### 2.1. Animals Group Treatment

A total of 25 male Wistar rats weighing between 240 and 250 g (aged 7 weeks) were from the Experimental Animal Center of Southern Medical University (Guangzhou, China). All rats were housed in static cages with controlled ambient temperature (22–25°C) on a 12-h light/dark cycle. After 1 week of acclimatization, the animals were randomly assigned to four groups: the control group (C) and iron overload group (IO) were fed with normal pellet diet (NPD) and five doses of intraperitoneal injection of 60 mg/kg iron-dextran-saline (ferric hydroxide dextran complex; Sigma, St. Louis, MO, USA) as previously described [22]. The T2D (D) and iron overload-related T2D (DIO) group were fed with the high-fat diet and injected with 35 mg/kg streptozotocin (STZ; Sigma, St. Louis, MO, USA) in the 4th week. For DIO group, the iron-dextran-saline was administrated with iron dextran saline, the same as IO group. The rats in all groups were weighed each week, and they were euthanized under ether anesthesia at 10 weeks after STZ injection. Before killing the rats, the blood glucose levels were measured by glucose test strips (Roche Diagnostic, Indianapolis, IN, USA). All protocols of animals and experiments were checked and appropriated by Animal Research Ethical Committee of Kunming University of Science and Technology (Kunming, China).

### 2.2. Determination of Glycolic Levels

On the 6th week and the last day of the treatment, the blood glycolic levels were measured to determine the success of diabetes induction using fresh blood with glucose test strips (Roche Diagnostics) according to the manufacturer's protocol.

### 2.3. Iron Parameters in Serum

Serum iron concentrations and total iron-binding capacity (TIBC) in nonhemolyzed serum samples were made by colorimetric analysis kits (Nanjing Jian Cheng Biotechnology Institute, Nanjing, China). In addition, serum ferritin was determined in nonhemolyzed serum samples using ELISA kits (Shanghai Enzyme-linked Biotechnology Co., Ltd., Shanghai, China).

### 2.4. Terminal Dexynucleotidyl Transferase-Mediated dUTP Nick End Labeling (TUNEL) Assay

According to the manufacturer's protocol, we have used TUNEL assay kit (Beyotime Company, Shanghai, China) for evaluating levels of cell apoptosis. Initially, every cell was fixed in 4% paraformaldehyde and permeabilized using 0.1% Triton X-100, and this process is repeated for every cell. After that, the cells were incubated in TUNEL reaction mixture for 1 h at 37°C. Nuclei were counterstained with DAPI, and the cells were observed with a Nikon Eclipse 80i microscope (Nikon, Tokyo, Japan).

### 2.5. Cell Culture and DIO Treatment

The rat INS-1 cells were purchased from Beijing Beina Chuanglian Biotechnology Institute (Beijing, China). Cells were cultured in RPMI1640 (Thermo Scientific, Waltham, MA, USA) containing 10% fetal bovine serum (Gibco; Thermo Fisher Scientific, Inc.), 50 *µ*M *β*-mercaptoethanol, and 1% penicillin and streptomycin (Gibco). Cells were incubated in a humidified atmosphere containing 5% CO_2_ at 37°C [23]. The medium was renewed once per two days, and cells were passaged once per 6 to 7 days. INS-1 cells in the logarithmic growth phase were used for the following tests. The control cells (NC) were cultured with 25 mmol/L glucose, which were treated with 12.5, 25, 50, 100, or 200 *μ*M iron-D for 48 h, respectively. At the end of the experiments, cell viability was determined.

### 2.6. Cell Transfection

Transfections were performed using miR-130a-3p mimic, miR-130a-3p inhibitor, and miRNA negative control, which were obtained from Shanghai GenePharma (Shanghai, China). The XIST and activin receptor-like kinase 2 (ALK2) overexpression vector (pc-XIST and pc-ALK2, respectively) were constructed to promote the expression of XIST and ALK2 in INS-1 cells, and the empty vector was used as a control. The XIST small interfering RNA was used to knock XIST expression. Cell transfection with the miRNA mimic, miRNA inhibitor, vectors, and siRNA was performed by using Lipofectamine 3000 (Invitrogen, Carlsbad, USA) according to the manufacturer's protocol.

### 2.7. Real-Time Quantitative PCR Analysis (RT-qPCR)

In these experiments, total RNA was extracted with TRIzol solution (Takara Biotechnology Co., Ltd., Dalian, Liaoning Province, China) and subsequently converted to cDNA with Reverse Transcription Kit (Takara) according to manufacturer's instruction. The levels of XIST, miR-130a-3p, GAPDH, and U6 were determined using SYBR Premix Ex TaqTM II kit (TaKaRa) and SYBR Premix Ex Taq miRNA kit (TaKaRa). The relative expression of XIST and miR-130a-3p was calculated using 2^−ΔΔCt^ method [24], whereas GAPDH and U6 were used as the reference gene.

### 2.8. Western Blot

Proteins were extracted, and the concentration was determined according to standard protocols of protein extraction and BCA protein assay kits, respectively (Sangon Biotech, Shanghai, China). The total protein in the supernatants (30 *μ*g/well) was separated by 10% SDS-PAGE and then transferred to PVDF membranes. After blocking with 5% skim milk, the membranes were incubated overnight at 4°C with anti-hepcidin (1 : 5000; no. ab190775, Abcam, Cambridge, MA, USA), anti-TfR1 (1 : 5000; no. ab269514, Abcam), anti-Ferritin (1 : 5000; no. ab75973, Abcam), anti-DMT1 (1 : 1000; no. ab157208, Abcam), anti-ALK2 (1 : 500; no. ab262699, Abcam), anti-BMP6 (1 : 1000; no. ab155963, Abcam), anti-SMAD1/5/8 (1 : 1000; orb162781, Biorbyt, UK), and anti-GAPDH (1 : 5000; no. ab8245, Abcam) antibodies. After three washes with TBST, the immunoblots were incubated with alkaline phosphatase-labeled goat anti-rabbit antibodies (1 : 1000, Cell Signaling Technology, USA). The immunoreactive bands were visualized using an enhanced chemiluminescence reagent (Sangon Biotech). The blots were semiquantified by ImageJ software 1.47 (National Institutes of Health, Bethesda, MD, USA).

### 2.9. Cell Viability Analysis

The viability of INS-1 cells was detected by using MTT kits (Sangon Biotech). Briefly, INS-1 cells were with RPMI-1640 and seeded into 96-well plates (2000 cells/well). The plate was incubated for 24 hours in a humidified incubator. 10 *μ*L MTT reagent was added at particular time points for 4 h at 37°C. The optical density (OD) was measured at 570 nm with a micrometer reader (BioTek Instruments Inc.).

### 2.10. Glucose Stimulated Insulin Secretion (GSIS) Assay

INS-1 cells were incubated in KRBH buffer (119 mM NaCl, 4.74 mM KCl, 1.20 mM KH2PO4, 1.19 mM MgSO_4_, 10 mM HEPES, 2.54 mM CaCl_2_, 25 mM NaHCO_3_, and 0.1% bovine serum albumin) containing 25 mmol/L concentrations of glucose for 1 h. The supernatants were centrifuged at 3000 rpm for 3 min, and then the insulin concentration was measured with ELISA kit (Abcam).

### 2.11. Labile Iron Pool (LIP) Evaluation

As previously described, cellular content of LIP-Fe was measured by fluorospectrophotometry using calcein-AM ester [25]. Briefly, INS-1 cells were seeded in 96-well plates and washed twice with phosphate-buffered saline (PBS) and incubated with calcein-AM (0.25 mmol/L) for 30 min at 37°C, whereas the fluorescence intensity was measured by fluorospectrophotometer (Ex = 495 nm, Em = 530 nm) using IPP 6.0 software package. Following the incubation in the medium-containing desferrioxamine (DFO, 100 mmol/L) for 30 min at 37°C, the fluorescence intensity was measured again. The LIP was calculated as the difference in calcein-AM cells treated with or without DFO. The increased LIP level of hepatocytes following various treatments was expressed as fold change over control.

### 2.12. Haematoxylin and Eosin (H&E) Staining

Pancreata tissues from each group rats were fixed in 10% neutral buffered formalin and processed for routine histology and paraffin embedding. Five micrometer tissue sections were stained with H&E and evaluated histologically to determine the degree of islet destruction. Staining of Brn3a was observed by Nikon Eclipse 80i microscope (Nikon Corporation).

### 2.13. Immunohistochemistry

The tissue sections were baked and deparaffinized. Antigen retrieval was performed by boiling in sodium citrate buffer. After blocking endogenous peroxidase and nonspecific binding, tissue sections were incubated with primary (anti-insulin, no. ab181547, Abcam) and then with secondary (no. ab150077, Abcam) antibody. The sections were washed (3 times), and the reaction product was developed with diamino benzoate, counterstained with hematoxylene. Staining of Brn3a was observed by Nikon Eclipse 80i microscope (Nikon Corporation).

### 2.14. Luciferase Reporter Assays

StarBase online software is used to predict the targeted binding sites of miRNAs in mRNAs and lncRNA. Here, we have predicted that the targeted binding relationships between miR-130a-3p and XIST or ALK2. We constructed reporter vectors, including wild-type (WT) and mutant-type (MUT) binding sites of XIST or ALK2 sequences, named as WT-XIST, MUT-XIST, WT-ALK2, and MUT-ALK2 and cotransfected with miR-130a-3p mimic or negative control into HEK 923 cells (ATCC, Manassas, VA, USA). Relative luciferase activity was assayed 48 h after transfection using the Dual-Luciferase reporter assay system (Promega Corporation, Wisconsin, USA).

### 2.15. Statistical Analysis

The data were expressed as mean ± standard error mean (SEM) and analyzed using Prism 8.0 (GraphPad Software Inc., San Diego, CA, USA). Data between the two groups were analyzed by Student's *t*-test, and data among multiple groups were analyzed by one-way analysis of variance (ANOVA) with Dunnet's least significant difference post-hoc tests. *P* < 0.05 was regarded as statistically significant. The results were considered significant when *P* < 0.05.

## 3. Results and Discussion

### 3.1. Effect of Iron Overload on Body Weight, Fasting Blood Glucose, Iron Parameters, and Pancreatic Islets/Beta Cells in T2D Rats

Compared with rats in the control group (NC), the individuals in T2D group (D) and iron overload-related T2D group (DIO) profiles had decreased body weights, while iron dextran injection only (IO) group showed no difference (Figure 1(a)). After 10th week, the weight gain of DIO group is slower than D group. Moreover, in D and DIO groups, rats performed a higher fasting blood glucose, and a more growth postprandial was observed (Figure 1(b)). To evaluate serum iron status, the serum iron and ferritin constituent and TIBC were measured. As shown in Figures 1(c)–1(e), three indexes were increased in IO and DIO groups. Next, the iron metabolic-related proteins were measured by Western blot, and results indicated that iron dextran-induced increased hepcidin, ferritin, and DMT1 proteins expression (Figure 1(f)). By contrast, the expression of TfR1 was decreased. Pancreatic morphology was analyzed to assess pathological changes. H&E staining revealed the well-defined islets of Langerhans, along with intact exocrine pancreatic tissues in control and IO groups, which were slightly lost in the sections from D group but seriously lost in the sections from DIO group (Figure 1(g), H&E staining). Sections of control and IO groups revealed dense reddish brown cytoplasmic immunoreactivity that was detected in the cells of the pancreatic islets of Langerhans. The immunoreactivity was observed in most of the islet cells (Figure 1(g), insulin staining). Sections of D group revealed slightly increased immunoreactivity, but sections of DIO group revealed markedly decreased immunoreactivity that was detected in the central part of the islet of Langerhans. Finally, we detected the expression of XIST in different groups, and results showed that the level of XIST was significantly increased in pancreas tissues as well as the pancreas of DIO compared with D group (Figure 1(h)). Notably, iron overload-induced promoted XIST expression in T2D.

### 3.2. XIST Is Involved in Iron Overload-Induced INS-1 Cells Injury

To further verify that lncRNA XIST was regulated by iron overload *in vitro*, INS-1 cells were treated with 12.5, 25, 50, 100, or 200 *μ*M iron-D for 48 h. As shown in Figure 2(a), iron-D reduced the survival of INS-1 cells in a concentration-dependent manner. The 50 *μ*M iron-D markedly reduced the survival of the INS-1 cells. Hence, cells treated with 50 *μ*M iron-D were used in the following study. To further explore the functions of XIST in INS-1 cells, we knocked the XIST in DIO cells (Figure 2(b)). Then, the result of MTT assay demonstrated that knockdown of XIST significantly promoted cell proliferation (Figure 2(c)). The TUNEL assay showed that the apoptotic cell in XIST knockdown group was less than that in DIO + sh-NC group (Figure 2(d)). Next, we tested that the iron overload decreased glucose-stimulated insulin secretion, and we found that compared with DIO + sh-NC group, knockdown of XIST could lighten the iron overload-related functional damage on INS-1 cells (Figure 2(e)). The LIP was upregulated in DIO, which was reserved by knockdown of XIST (Figure 2(f)). Furthermore, we detected whether XIST affected the iron metabolic-related proteins, and results indicated that XIST knockdown could downregulate the expression of hepcidin, ferritin, and DMT1 but upregulated TfR1 expression (Figure 2(g)). These findings showed that XIST may influence the iron metabolism and is involved in iron overload-induced islet beta cells injury.

### 3.3. XIST Targets and Regulates miR-130a-3p

Targeting miRNA is one of the regulatory functions of lncRNA. The StarBase predicted that XIST contained complementary binding sites to miR-130a-3p (Figure 3(a)). In previous studies, XIST may act as a competitive endogenous RNA (ceRNA) by inhibiting miR-130a-3p. Hence, we speculated that there is targeting relationship between XIST and miR-130a-3p. To confirm it, a fragment of XIST including the putative WT or MUT binding sites was constructed into the luciferase reporter vectors. As shown in Figure 3(b), the cotransfection with the miR-130a-3p mimics and XIST-WT resulted in an obvious decrease of luciferase activity in HEK 923 cells, while no significant effect was present in cell transfected with the miR-130a-3p mimics and XIST-MUT. Overexpression of XIST markedly decreased miR-130a-3p expression (Figure 3(c)). Interestingly, we found miR-130a-3p expressed less in rats and INS-1 cells of DIO group, and sh-XIST markedly increased miR-130a-3p expression (Figures 3(d) and 3(e)). Taken together, XIST directly targets miR-130a-3p.

### 3.4. XIST Increases Iron Overload-Induced INS-1 Cells Injury by Targeting miR-130a-3p

To further investigate the regulatory network of XIST and miR-130a-3p, the miR-130a-3p mimics and pc-XIST were cotransfected into INS-1 cells. As shown in Figure 4(a), miR-130a-3p mimics transfection upregulated miR-130a-3p levels, while XIST overexpression significantly decreased the expression of miR-130a-3p in cotransfected group. Additionally, miR-130a-3p overexpression promoted proliferation and inhibited apoptosis of INS-1 cells (Figures 4(b) and 4(c)). More than that, XIST overexpression reversed the effects of miR-130a-3p overexpression on proliferation and apoptosis of INS-1 cells. The insulin secretion in miR-130a-3p overexpression was higher than that in both NC group and miR-130a-3p mimics + pc-XIST groups (Figure 4(d)). The LIP was downregulated in overexpression of miR-130a-3p, which was reserved by XIST upregulation (Figure 4(e)). Furthermore, overexpression of miR-130a-3p increased the level of hepcidin, ferritin, and DMT1 proteins, inhibited by overexpression of XIST (Figure 4(f)). By contrast, overexpression of miR-130a-3p decreased TfR1 protein level but was reversed by upregulation of XIST. These findings demonstrated that high expression of miR-130a-3p protects islet beta cells from iron overload, which is reversed by overexpression of XIST.

### 3.5. ALK2 Is a Target mRNA of miR-130a-3p

ALK2 has been demonstrated to be a direct target of miR-130a [26]. As shown in Figure 5(a), ALK2 mRNA harbored the binding site of miR-130a-3p. The effects of iron overload, XIST, and miR-130a-3p on ALK2 expression are elucidated. Then, we detected the protein level of ALK2 in the animal model and found that ALK2 was upregulated in D and DIO groups compared with the control and IO groups, and DIO group was higher compared with D group (Figure 5(b)). Furthermore, ALK2 expression was inhibited and promoted by miR-130a-3p inhibitors and miR-130a-3p mimics, respectively, while cotransfection with miR-130a-3p mimics and pc-XIST had no significant influence on the protein level of ALK2 (Figure 5(c)). The result of luciferase assay showed that compared with the control group, the luciferase activity was significantly decreased in cell cotransfected with ALK2-WT and miR-130a-3p mimics, while that in cotransfected ALK2-MUT and miR-130-3p mimics did not significantly change (Figure 5(d)). Taken together, miR-130a-3p directly targeted ALK2.

### 3.6. XIST Promotes Iron Overload-Induced INS-1 Cells Injury by Regulating miR-130a-3p/ALK2 Axis

To explore the function of XIST/miR-130a-3p/ALK2 axis in iron overload, the miR-130a-3p mimic, pc-XIST, and sh-ALK2 were cotransfected into INS-1 cells. The expression of ALK2 was reduced by interference of ALK2, which was revered with overexpression of XIST, but ALK2 expression was finally repressed by miR-130a-3p mimics (Figure 6(a)). On the contrary, cell proliferation and survival rate were elevated after interference of ALK2 but reduced with XIST upregulation, which was terminally boosted by miR-130a-3p mimics (Figures 6(b) and 6(c)). Next, the LIP and insulin secretion were measured, as shown in Figures 6(d) and 6(e), respectively. The results indicated that downregulation of ALK2 lowered LIP, which was revered with XIST overexpression but LIP was finally decreased by miR-130a-3p upregulation (Figure 6(d)). On the contrary, insulin secretion was increased after ALK2 knockdown but decreased with XIST upregulation, which was terminally boosted by miR-130a-3p upregulation (Figure 6(e)). These results suggest that XIST/miR-130a-3p/ALK2 axis regulates islet beta cells injury from iron overload.

It is well established that hepcidin has emerged as the key regulator of uptake and release of iron in the tissues and cells [27]. Bone morphogenetic protein 6 (BMP6) binds to the ALK2 and AKL3 from a heterodimeric complex previously reported to increase hepcidin transcription expression by inducing phosphorylation of SMAD1/5/8 [26]. Therefore, we explored whether ALK2 modulated BMP6/AMAD signaling in iron metabolic. The levels of BMP6 and p-SMAD1/5/8 were decreased after knockdown of ALK2 but were increased with overexpression of XIST, which was terminally repressed by miR-130a-3p upregulation (Figure 6(f)). These results confirmed the ALK2 positive regulation of BMP6/AMAD signaling. Next, iron metabolic-related proteins level was measured by using Western Blot. The expressions of hepcidin and DMT1 were reduced by interference of ALK2, which were revered with overexpression of XIST, but hepcidin and DMT1 expression were finally repressed by miR-130a-3p upregulation (Figure 6(f)). On the contrary, the expression of TfR1 was elevated after interference of ALK2 but reduced with XIST upregulation, which was terminally boosted by miR-130a-3p overexpression. These results suggest that XIST/miR-130a-3p/ALK2 axis may protect islet beta cells from iron overload by BMP6/AMAD signaling.

### 3.7. Knockdown of XIST Alleviates Iron Overload-Induced Pancreatic Islets/Beta Cells Injury in T2D Rats

To determine the role of XIST in iron overload-induced pancreatic islets/beta cells, we silenced XIST expression in the DIO rats (Figure 7(a)). Notably, XIST depletion significantly increased and decreased the expression of miR-130a-3p and ALK2, respectively (Figures 7(b) and 7(c), respectively). Additionally, XIST knockdown remarkably alleviated iron overload-induced body weight loss (Figure 7(d)). By contrast, XIST knockdown significantly inhibited iron overload-induced blood glucose, serum iron, TIBC, and serum ferritin levels rise (Figures 7(e)–7(h), respectively). The protein expressions of BMP6, SMAD1/5/8, hepcidin, ferritin, and DMT1 were elevated by iron overload-induced but was reversed with knockdown of XIST (Figure 7(i)). On the contrary, TfR1 protein expression was reduced after iron overload-induced, which was reversed with XIST knockdown. H&E staining revealed the well-defined islets of Langerhans, along with intact exocrine pancreatic tissues in control group, seriously lost in DIO group (Figure 7(j), H&E staining). Sections of control group revealed dense reddish brown cytoplasmic immunoreactivity, which was markedly decreased (Figure 7(j), insulin staining). There was an improvement in the histology of pancreatic and insulin secretion from XIST knockdown treated groups. These data indicate that XIST knockdown alleviates iron overload-induced pancreatic islets/beta cells injury in T2D rats.

## 4. Discussion

Iron is an essential element, but the iron deposition will result in the reduction of the number of islet beta cells and insulin secretion as described in [28], thus, promoting the occurrence and development of diabetes mellitus [29]. In this study, we have shown that iron overload promoted weight loss and increase of postprandial blood glucose by increasing the expression of iron, TIBC, ferritin, hepcidin, and DMT1 and decreasing the expression of TfR1. Through RT-qPCR analysis, we identified XIST upregulated in T2D. Notably, iron overload did not affect XIST expression but promoted XIST expression in T2D. These observations suggest that XIST plays a critical role in the iron metabolism of T2D.

LncRNAs have been reported to play widespread roles in gene regulation and other cellular processes [30]. LncRNAs exert their functions via diverse mechanisms, including cotranscriptional regulation, modulation of gene expression, scaffolding of nuclear or cytoplasmic complexes, and pairing with other RNAs [31]. Notably, accumulating evidence shows that lncRNAs are implicated in T2D [32] and iron overload [33]. XIST was highly expressed in T2D patients [18] and was activated by iron overload. Aberrant expression of XIST is implicated in diabetes mellitus and its complications [18, 34, 35]. Here, we show that knockout of XIST expression impairs the iron overload-induced injury and iron metabolism of INS-1 cells, suggesting that XIST-medicated iron metabolism is critical for iron overload-induced islet beta cells injury.

Studies have shown that lncRNAs can serve as a miRNA ceRNA regulatory network in many diseases [36]. For example, lncRNA ROR could serve as a ceRNA, which regulates islet beta cell differentiation by sponging miR-145 to target Sox2 [37]. In this study, we found that miR-130a-3p was downregulated and determined as a target of XIST and negatively regulated by XIST, thereby inhibiting iron overload and iron overload-induced injury of INS-1 cells. According to reports, miR-130a is upregulated in mouse liver by iron deficiency and targets the BMP receptor ALK2 to attenuate BMP signaling and hepcidin transcription [26]. Interestingly, miR-130a-3p is upregulated in iron deficiency and downregulated in iron overload, suggesting that iron dose regulates miR-130a-3p expression. However, in this study, upregulation of miR-130a-3p changed iron metabolism and ameliorated iron overload-induced INS-1 cells injury. Recent studies reported that miR-130a-3p is lowly expressed in diabetes mellitus and its complications, and upregulation of miR-130a-3p ameliorates the unhealthy condition of renal tubular epithelial and pancreatic beta cells [38, 39]. Thus, we identified miR-130a-3p as an efficient regulator of iron metabolism in T2D.

Furthermore, the miR-130a-3p and its target gene ALK2 were identified as the downstream molecule of XIST. Our findings revealed that the role of XIST/miR-130a-3p/ALK2 axis regulated iron overload and played a role in T2D pathology. ALK2 (also known as ACVR1) is a BMP type-I receptor subtype that plays an important physiological role in the development of bones, muscles, brain, and other organs [40]. BMP6 binds to the ALK2 and ALK3 from a heterodimer complex to increase hepcidin transcription expression by inducing phosphorylation of SMAD1/5/8 [26]. Hepcidin has emerged as the key regulator of uptake and release of iron in the tissues and cells, suggesting that ALK2 plays a critical role in iron metabolism. MiR-130a is upregulated in mouse liver by iron deficiency and attenuates BMP signaling and hepcidin transcription by targeting ALK2 [26]. Here, we found that XIST can sponge miR-130a-3p to trigger ALK2 expression, leading to the priming of INS-1 cells iron overload. Knockdown of BMP6 and its receptors ALK2/3/6 with siRNA decreases hepcidin transcription [41]. We also found that knockdown of ALK2 promoted iron transport by decreasing hepcidin transcription via inhibited SMAD1/5/8 activation. Interestingly, BMP6 is the primary upstream gene of ALK2 but BMP6 expression was decreased by knocking ALK2 expression, which also was subjected to the feedback regulation of its downstream signaling in T2D. Therefore, the feedback regulation in iron overload remains to be further investigated.

## 5. Conclusion

In this paper, we have proposed a novel approach and verified its applicability through various experiments. The results showed that XIST overexpression in iron overload rats was associated with a coincident alteration in iron-related parameters. *In vitro*, increasing XIST level in response to iron-induced was associated with iron metabolism, proliferation inhibition, apoptosis, and reduction of insulin secretion. In contrast, XIST knockdown alleviated above islet *β*-cell damage induced by iron overload. XIST can promote islet beta cells iron overload and T2D initiation and development through inhibition of ALK2 expression by sponging miR-130a-3p. Our findings reveal that XIST/miR-130a-3p/ALK2 axis may play a crucial role in the progression of T2D and that targeting this axis may be an effective strategy for treating patients with T2D.

## Figures and Tables

**Figure 1:** XIST is less expressed in iron-related T2D model. NC = citrate control (*n* = 5); D = diabetes (*n* = 5); IO = iron overload (*n* = 5); DIO = diabetes/iron overload (*n* = 5). (a) The body weight of control group, iron overload group, T2D model group, and iron overload related T2D group rats. (b) Comparison of postprandial and fasting blood glucose concentration in serum. ((c), (d), (e)) Comparison of iron, TIBC, and ferritin constituent in serum. (f) Comparison of iron metabolic-related proteins of differently treated rats. (g) The H&E and insulin staining in pancreatic tissues. Scale bar = 100 *μ*m. (h) Comparison of XIST level pancreas tissues from rats, respectively. ^*∗*^*P* < 0.05, ^*∗∗*^*P* < 0.01.

**Figure 2:** XIST knockdown alleviates the iron overload-induced damage on INS-1 cells. (a) INS-1 cells were treated with different concentrations of iron-D. (b) The expression of XIST in islet beta cells transfected with control, vector, and sh-XIST detected by RT-qPCR. (c) Cell proliferation after transfection at different times was measured by MTT assay. Scale bar = 100 *μ*m. (d) Representative results of TUNEL staining for every group. (e) GSIS assay was used to measure the secretion of insulin. (f) Knockdown of XIST downregulated LIP. (g) The protein expressions of hepcidin, TfR1, ferritin, and DMT1 in INS-1 cells were measured by Western blot. ^*∗*^*P* < 0.05, ^*∗∗*^*P* < 0.01.

**Figure 3:** XIST directly binds to and regulates the expression of miR-130a-3p. (a) The predicted binding sites of miR-130a-3p to XIST sequence using StarBase. (b) The relative luciferase of HEK 923 cells was transfected with miR-130a-3p mimics and luciferase constructs of wild-type (WT) or mutated-type (MUT) XIST-UTR. (c) Overexpression of XIST decreased miR-130a-3p expression. (d) The expression level of miR-130a-3p in tissues of rat. (e) The expression level of miR-130a-3p in INS-1 cells. ^*∗∗*^*P* < 0.01.

**Figure 4:** XIST reversed the protective effects of miR-130a on INS-1 cells. (a) The expression of miR-130a-3p in INS-1 cells transfected with control, vector, miR-130a-3p mimics, and pc-XIST detected by RT-qPCR analysis. (b) Cell proliferation after transfection different time was measured by MTT assay. (c) Representative results of TUNEL staining for every group. Scale bar = 100 *μ*m. (d) GSIS was used to measure the secretion of insulin. (e) The LIP level was detected for every group. (f) The iron metabolic-related protein expression was detected in islet beta cells. ^*∗*^*P* < 0.05, ^*∗∗*^*P* < 0.01.

**Figure 5:** miR-130a-3p directly binds to and regulates the expression of ALK2. (a) The predicted binding sites of miR-130a-3p to ALK2 sequence using StarBase. ((b) and (c)) The expression of ALK2 protein was detected by Western blot. (d) The relative luciferase of HEK 923 cells was transfected with miR-130a-3p mimics or inhibitors and luciferase constructs of WT- or MUT-ALK2-UTR. ^*∗∗*^*P* < 0.01.

**Figure 6:** XIST promotes iron overload-induced INS-1 cells injury by regulating miR-130a-3p/ALK2 axis. (a) The expression of ALK2 protein was detected by Western blot. (b) Cell proliferation was measured by MTT assay. (c) Representative results of TUNEL staining for every group. Scale bar = 100 *μ*m. (d) Knockdown of XIST downregulated LIP. (e) GSIS assay was used to measure the secretion of insulin. (f) The protein expression was measured by Western blot. ^*∗*^*P* < 0.05, ^*∗∗*^*P* < 0.01.

**Figure 7:** Knockdown of XIST alleviates iron overload-induced pancreatic islets/beta cells injury in T2D rats. ((a) and (b)) The gene expression was detected by RT-qPCR. (c) The expression of ALK2 protein was detected by Western blot. (d) The body weight of each group rats. (e) Comparison of postprandial and fasting blood glucose concentration of differently treated rats. ((f), (g), (h)) Comparison of iron, TIBC, and ferritin constituent in serum from each group. (i) Comparison of iron metabolic-related proteins of differently treated rats. (j) The H&E and insulin staining in pancreatic tissues. Scale bar = 100 *μ*m. ^*∗*^*P* < 0.05, ^*∗∗*^*P* < 0.01.

## Data Availability

The datasets used and analyzed during the current study are available from the corresponding author upon reasonable request.

## References

[1] Warr C. G., Shaw K. H., Azim A., Piper M. D. W., Parsons L. M. (2018). Using mouse and Drosophila models to investigate the mechanistic links between diet, obesity, type II diabetes, and cancer. *International Journal of Molecular Sciences*.

[2] Zaccardi F., Webb D. R., Yates T., Davies M. J. (2016). Pathophysiology of type 1 and type 2 diabetes mellitus: a 90-year perspective. *Postgraduate Medical Journal*.

[3] Aldersley M. A., Allgar V., Howdle P. D., Markham A. F. (1998). Haemochromatosis and type 2 diabetes. *The Lancet*.

[4] Kishimoto M., Endo H., Hagiwara S., Miwa A., Noda M. (2010). Immunohistochemical findings in the pancreatic islets of a patient with transfusional iron overload and diabetes: case report. *Journal of Medical Investigation*.

[5] Simcox J. A., McClain D. A. (2013). Iron and diabetes risk. *Cell Metabolism*.

[6] Kataria Y., Wu Y., Horskjær P., Mandrup-Poulsen T., Ellervik C. (2018). Iron status and gestational diabetes-A meta-analysis. *Nutrients*.

[7] Wilman H. R., Parisinos C. A., Atabaki-Pasdar N. (2019). Genetic studies of abdominal MRI data identify genes regulating hepcidin as major determinants of liver iron concentration. *Journal of Hepatology*.

[8] Sachinidis A., Doumas M., Imprialos K., Stavropoulos K., Katsimardou A., Athyros V. G. (2020). Dysmetabolic iron overload in metabolic syndrome. *Current Pharmaceutical Design*.

[9] Li D., Jiang C., Mei G. (2020). Quercetin alleviates ferroptosis of pancreatic *β* cells in type 2 diabetes. *Nutrients*.

[10] Kullmann S., Heni M., Hallschmid M., Fritsche A., Preissl H., Häring H. U. (2016). Brain insulin resistance at the crossroads of metabolic and cognitive disorders in humans. *Physiological Reviews*.

[11] Fernández-Real J. M., McClain D., Manco M. (2015). Mechanisms linking glucose homeostasis and iron metabolism toward the onset and progression of type 2 diabetes. *Diabetes Care*.

[12] Varghese J., James J. V., Anand R. (2020). Development of insulin resistance preceded major changes in iron homeostasis in mice fed a high-fat diet. *Journal of Nutritional Biochemistry*.

[13] Morris K. V., Mattick J. S. (2014). The rise of regulatory RNA. *Nature Reviews Genetics*.

[14] Jain S., Thakkar N., Chhatai J., Pal Bhadra M., Bhadra U. (2017). Long non-coding RNA: functional agent for disease traits. *RNA Biology*.

[15] Morán I., Akerman I., van de Bunt M. (2012). Human *β* cell transcriptome analysis uncovers lncRNAs that are tissue-specific, dynamically regulated, and abnormally expressed in type 2 diabetes. *Cell Metabolism*.

[16] Ding G. L., Wang F. F., Shu J. (2012). Transgenerational glucose intolerance with Igf2/H19 epigenetic alterations in mouse islet induced by intrauterine hyperglycemia. *Diabetes*.

[17] Wu Y., Huang C., Meng X., Li J. (2015). Long noncoding RNA MALAT1: insights into its biogenesis and implications in human disease. *Current Pharmaceutical Design*.

[18] Sathishkumar C., Prabu P., Mohan V., Balasubramanyam M. (2018). Linking a role of lncRNAs (long non-coding RNAs) with insulin resistance, accelerated senescence, and inflammation in patients with type 2 diabetes. *Human Genomics*.

[19] Chen K., Ma Y., Wu S. (2019). Construction and analysis of a lncRNA-miRNA-mRNA network based on competitive endogenous RNA reveals functional lncRNAs in diabetic cardiomyopathy. *Molecular Medicine Reports*.

[20] Yang J., Shen Y., Yang X. (2019). Silencing of long noncoding RNA XIST protects against renal interstitial fibrosis in diabetic nephropathy via microRNA-93-5p-mediated inhibition of CDKN1A. *American Journal of Physiology - Renal Physiology*.

[21] Xu Y., Luo X., He W. (2018). Long non-coding RNA PVT1/miR-150/HIG2 Axis regulates the proliferation, invasion and the balance of iron metabolism of hepatocellular carcinoma. *Cellular Physiology and Biochemistry*.

[22] Zhang Y., Huang Y., Deng X., Xu Y., Gao Z., Li H. (2012). Iron overload-induced rat liver injury: involvement of protein tyrosine nitration and the effect of baicalin. *European Journal of Pharmacology*.

[23] He C., Zheng X., Lin X., Chen X., Shen C. (2020). Yunvjian-medicated serum protects INS-1 cells against glucolipotoxicity-induced apoptosis through autophagic flux modulation. *Evidence-based Complementary and Alternative Medicine*.

[24] Livak K. J., Schmittgen T. D. (2001). Analysis of relative gene expression data using real-time quantitative PCR and the 2−ΔΔCT method. *Methods*.

[25] Li Y., Deng Y., Tang Y. (2014). Quercetin protects rat hepatocytes from oxidative damage induced by ethanol and iron by maintaining intercellular liable iron pool. *Human & Experimental Toxicology*.

[26] Zumbrennen-Bullough K. B., Wu Q., Core A. B. (2014). MicroRNA-130a is up-regulated in mouse liver by iron deficiency and targets the bone morphogenetic protein (BMP) receptor ALK2 to attenuate BMP signaling and hepcidin transcription. *Journal of Biological Chemistry*.

[27] Agarwal A. K., Yee J. (2019). *Advances in Chronic Kidney Disease*.

[28] Shu T., Lv Z., Xie Y., Tang J., Mao X. (2019). Hepcidin as a key iron regulator mediates glucotoxicity-induced pancreatic *β*-cell dysfunction. *Endocrine Connections*.

[29] Ambachew S., Biadgo B. (2017). Hepcidin in iron homeostasis: diagnostic and therapeutic implications in type 2 diabetes mellitus patients. *Acta Haematologica*.

[30] Wang K. C., Chang H. Y. (2011). Molecular mechanisms of long noncoding RNAs. *Molecular Cell*.

[31] Ponting C. P., Oliver P. L., Reik W. (2009). Evolution and functions of long noncoding RNAs. *Cell*.

[32] He X., Ou C., Xiao Y., Han Q., Li H., Zhou S. (2017). LncRNAs: key players and novel insights into diabetes mellitus. *Oncotarget*.

[33] Wróblewska A., Bernat A., Woziwodzka A. (2017). Interferon lambda polymorphisms associate with body iron indices and hepatic expression of interferon-responsive long non-coding RNA in chronic hepatitis C. *Clinical and Experimental Medicine*.

[34] Long B., Wan Y., Zhang S., Lv L. (2020). LncRNA XIST protects podocyte from high glucose-induced cell injury in diabetic nephropathy by sponging miR-30 and regulating AVEN expression. *Archives of Physiology and Biochemistry*.

[35] Yao D., Lin Z., Zhan X., Zhan X. (2020). Identifying potential functional lncRNAs in metabolic syndrome by constructing a lncRNA-miRNA-mRNA network. *Journal of Human Genetics*.

[36] Karreth F. A., Pandolfi P. P. (2013). ceRNA cross-talk in cancer: when ce-bling rivalries go awry. *Cancer Discovery*.

[37] Zou G., Liu T., Guo L. (2016). miR-145 modulates lncRNA-ROR and Sox2 expression to maintain human amniotic epithelial stem cell pluripotency and *β* islet-like cell differentiation efficiency. *Gene*.

[38] Ofori J. K., Salunkhe V. A., Bagge A. (2017). Elevated miR-130a/miR130b/miR-152 expression reduces intracellular ATP levels in the pancreatic beta cell. *Scientific Reports*.

[39] Jiang X., Ruan X. L., Xue Y. X., Yang S., Shi M., Wang L. N. (2020). Metformin reduces the senescence of renal tubular epithelial cells in diabetic nephropathy via the MBNL1/miR-130a-3p/STAT3 pathway. *Oxidative Medicine and Cellular Longevity*.

[40] Sekimata K., Sato T., Sakai N. (2020). ALK2: a therapeutic target for fibrodysplasia ossificans progressiva and diffuse intrinsic pontine glioma. *Chemical and Pharmaceutical Bulletin*.

[41] Luo X., Luo Z., Zhang Z. (2016). Homocysteine upregulates hepcidin expression through BMP6/SMAD signaling pathway in hepatocytes. *Biochemical and Biophysical Research Communications*.

